# VIP/PACAP-Based Drug Development: The ADNP/NAP-Derived Mirror Peptides SKIP and D-SKIP Exhibit Distinctive *in vivo* and *in silico* Effects

**DOI:** 10.3389/fncel.2019.00589

**Published:** 2020-01-14

**Authors:** Shlomo Sragovich, Noy Amram, Adva Yeheskel, Illana Gozes

**Affiliations:** ^1^The Lily and Avraham Gildor Chair for the Investigation of Growth Factors, The Elton Laboratory for Neuroendocrinology, Department of Human Molecular Genetics and Biochemistry, Sackler Faculty of Medicine, Sagol School of Neuroscience and Adams Super Center for Brain Studies, Tel Aviv University, Tel Aviv, Israel; ^2^Bioinformatics Unit, George S. Wise Faculty of Life Sciences, Tel Aviv University, Tel Aviv, Israel

**Keywords:** ADNP, NAP, SKIP, D-SKIP, VIP, PACAP, ASD

## Abstract

Activity-dependent neuroprotective protein (ADNP) was discovered and first characterized in the laboratory of Prof. Illana Gozes to be regulated by vasoactive intestinal peptide (VIP), and pituitary adenylate cyclase-activating peptide (PACAP) toward neuroprotection. Importantly, ADNP is a master regulator of >400 genes, essential for brain formation, while its haploinsufficiency causes cognitive impairments. Recently, *de novo* mutations in ADNP were identified as leading to the autism-like *ADNP* syndrome, mimicked by the *Adnp*-deficient mouse model. Furthermore, novel peptide derivatives of the neuroprotective ADNP-snippet NAP (NAPVSIPQ), developed in our laboratory, include SKIP and the mirroring all D-amino acid SKIP (D-SKIP). We now extended previous evidence suggesting potential antagonistic features for D-SKIP, compared with the neuroprotective peptide SKIP, as was observed by NMR analysis and social/olfactory functional testing. Here, an impact of the *Adnp* genotype was observed in the Morris Water Maze (MWM) test measuring cognition, coupled with improvement by SKIP, opposing the inert/exacerbating effect of D-SKIP. In the elevated plus-maze and open field tests measuring anxiety-related behaviors, contrasting effects of SKIP and D-SKIP were found, with SKIP improving/preserving the normal phenotype of the mouse, and D-SKIP causing alterations. Lastly, an *in silico* analysis suggested that SKIP and D-SKIP bind the microtubule end binding (EB) proteins EB1 and EB3 in different conformations, thereby indicating distinctive natures for the two peptides, potentially mediating differential *in vivo* effects. Altogether, our findings corroborate the notion of D-SKIP acting as an antagonist, thus distinguishing it from the neuroprotective SKIP.

## Introduction

Activity-dependent neuroprotective protein (ADNP) and activity-dependent neuroprotective factor (ADNF) were originally discovered and characterized in our laboratory (IG) in collaboration with the laboratory of Dr. Douglas E. Brenneman as astroglial secreted proteins, found to mediate the neurotrophic/neuroprotective activity of vasoactive intestinal peptide (VIP; Brenneman and Gozes, 1996; Bassan et al., 1999), as well as pituitary adenylate cyclase-activating peptide (PACAP; Zusev and Gozes, 2004). Importantly, ADNP is essential for mammalian brain formation (Bassan et al., 1999; Zamostiano et al., 2001; Pinhasov et al., 2003; Vulih-Shultzman et al., 2007), and function, as it was shown that complete knockout of the *Adnp* gene in mice results in embryonic lethality due to a failure in neural tube closure (Pinhasov et al., 2003). Nevertheless, *Adnp*-haploinsufficient mice (*Adnp*^+/–^) survive but exhibit cognitive and social deficits, as well as microtubule-tau pathology and neurodegeneration (Vulih-Shultzman et al., 2007), even when being outbred (Malishkevich et al., 2015; Amram et al., 2016; Hacohen-Kleiman et al., 2018), thus confirming the impact of ADNP on neuronal function and *in vivo* behavior.

Furthermore, the Gozes laboratory identified a small active 8-amino-acid peptide (NAPVSIPQ = NAP, also called davunetide or CP201), derived from ADNP. NAP was shown to enhance cognitive function in *Adnp*^+/–^ mice (Vulih-Shultzman et al., 2007; Hacohen-Kleiman et al., 2018; Sragovich et al., 2019a), by interacting with tubulin/microtubule end binding (EB) proteins through its SIP motif (NAPVSIPQ; Oz et al., 2014), eventually leading to microtubule stabilization and fortification (Gozes et al., 2005). Similarly, additional peptides developed in our lab were derived from ADNF, namely ADNF-14 (VLGGGSALLRSIPA) and ADNF-9 (SALLRSIPA = SAL), both sharing the SIP motif with NAP (Gozes et al., 2000b), and exhibiting neuroprotective activity (Brenneman and Gozes, 1996; Brenneman et al., 1998). Interestingly, both D- and L-amino acid forms of ADNF-9 (SAL) exhibited similar neuroprotective potency, with the D-amino acid form being protease stable and suitable for oral administration (Brenneman et al., 2004; Wilkemeyer et al., 2004; Parnell et al., 2007), further found to be neuroprotective *in vitro* and *in vivo* (Gozes et al., 2008; Shiryaev et al., 2011).

NAP safety and efficacy profiles were also translated to humans, showing favorable intranasal brain bioavailability, broad safety profile (Gozes et al., 2005), as well as cognitive and functional protection in clinical trials involving patients suffering from amnestic mild cognitive impairment and schizophrenia (Javitt et al., 2012; Jarskog et al., 2013; Morimoto et al., 2013a,b). Based on the SIP motif, serving as the NAP EB binding site, a NAP-derived 4-amino acid peptide, SKIP, was developed. This peptide contains only the EB-binding site, and was previously found to protect social memory, axonal transport, as well as correct hippocampal gene expression in the *Adnp*^+/–^ mouse model (Amram et al., 2016). In parallel, a dextrorotatory analog peptide, D-SKIP, was also developed in the lab, and further suggested to have an antagonistic activity, as was observed by NMR analysis and social/olfactory functional testing (Amram et al., 2016).

Recently, ADNP was found to be mutated *de novo* in 0.17% of autism spectrum disorder (ASD) cases, thus causing the *ADNP* syndrome. A thorough characterization of this pathologic condition has revealed cognitive deficits (Helsmoortel et al., 2014), global developmental delays, intellectual disabilities (ID), speech impediments and motor dysfunctions (Gozes et al., 2017a; Van Dijck et al., 2019). In this regard, the human *ADNP* syndrome patient was shown to be mimicked by the *Adnp*-haploinsufficient mouse model, implying a strong impact of the *Adnp* genotype, which included neurodevelopmental delays, as well as cognitive, social, and motor deficits (Hacohen-Kleiman et al., 2018). At the synapse level, reduced dendritic spine density and altered synaptic gene expression were also observed in *Adnp*-deficient mice. In terms of therapeutics, systemic/nasal administration of the drug candidate, NAP, provided improvement at all investigated levels spanning from synapse to behavior in *Adnp*^+/–^ mice (Hacohen-Kleiman et al., 2018). Therefore, these findings established the *Adnp*-haploinsufficient mouse as a valid model for the human *ADNP* syndrome patient and provided a solid basis for the further clinical development of NAP (CP201) in children suffering from the *ADNP* syndrome (Hacohen-Kleiman et al., 2018).

In the current article, we sought to characterize and provide additional evidence for the antagonistic nature of D-SKIP. For this purpose, the study involved male mice subjected to several *in vivo* behavioral tests including the Morris Water Maze (MWM) test measuring cognition, as well as elevated plus maze (EPM) and open field tests measuring anxiety-related behavior. Results showed cognitive impairments in *Adnp*^+/–^ mice, observed in the MWM test, coupled with improvement by SKIP treatment. In contrast, D-SKIP exhibited a distinctive effect, with an aggravated phenotype displayed in *Adnp*^+/+^ mice in the MWM, and with no amelioration observed in *Adnp*^+/–^ mice. Anxiety-related behavior assessed in the EPM and open field tests were improved/normally preserved by SKIP treatment in *Adnp*^+/+^ mice or remained unaffected in their *Adnp*^+/–^ counterparts. As opposed, D-SKIP-treated mice of both genotypes presented an altered phenotype. Lastly, *in silico* bioinformatics analysis showed that SKIP and D-SKIP bind EB1 and EB3 proteins in different conformations. Therefore, our present results provide further characterization/substantiation of D-SKIP as a potential antagonist, since D-SKIP did not mimic the SKIP effect. Furthermore, in some cases, D-SKIP acted as an inert compound not causing any effect, whereas in other cases it exacerbated the wildtype phenotype.

## Materials and Methods

### Experimental Design

Animal group sizes were determined in a pilot study, and animals were randomly allocated into experimental groups before the experiment. Blinded experienced researchers performed independently the different methodologies described in the manuscript, and repeated these successfully, thus substantiating the results. Biological replicates were used for all the *in vivo* procedures described in the manuscript. The exact experimental group allocations are included in each figure legend.

### Animals

The *Adnp*^+/–^ mice, on a mixed C57BL and 129/Sv background, were previously described (Pinhasov et al., 2003; Vulih-Shultzman et al., 2007). For continuous breeding, an ICR outbred mouse line was used (Malishkevich et al., 2015; Amram et al., 2016). Animals were housed in a 12-h light/12-h dark cycle animal facility, with free access to rodent chow and water. Genotyping was performed by Transnetyx (Memphis, TN, USA). Furthermore, for all *in vivo* behavioral procedures, animals were tracked, monitored and recorded using the EthoVision XT video tracking system and software (Noldus Inc., Leesburg, VA, USA). The MWM and open field *in vivo* tests were performed under bright illumination conditions (light levels of ~500 lux), whereas the elevated plus-maze was performed with a dim light.

### Peptide Synthesis and SKIP/D-SKIP Treatment

SKIP and D-SKIP were customarily synthesized by Hay Laboratories, Israel. Prior to beginning behavioral tests, intranasal treatment was administered twice daily, 5 days a week, over a 1-month period to 6-month-old male mice (2 μg/5 μl/mouse/dose), followed by a chronic daily administration regime of the peptides. For intranasal administration, the peptides were dissolved in a vehicle solution (Alcalay et al., 2004), termed DD, in which each milliliter included 7.5 mg of NaCl, 1.7 mg of citric acid monohydrate, 3 mg of disodium phosphate dihydrate, and 0.2 mg of benzalkonium chloride solution (50%). SKIP/D-SKIP or vehicle solution (DD) were administered to mice hand-held in a semi-supine position with nostrils facing the investigator. A pipette tip was used to administer 5 μl/mouse/dose. The mouse was handheld until the solution was totally absorbed (~10 s). In days of scheduled behavioral tests, SKIP/D-SKIP were applied once a day, 2 h before the test.

### Morris Water Maze (MWM)

The apparatus was a pool with a diameter of 140 cm, filled with opaque water (23–24°C). An escape platform (12 × 12 cm^2^) was placed 0.5 cm below the water surface. Two daily tests, constituting two blocks of trials, 90 s each, were performed for five consecutive days (Gozes et al., 2000a). The platform location and the animal starting point were held constant within each pair of daily tests, but they were changed from day-to-day. The mice were allowed to stay on the platform for 20 s before and after each trial. The time taken for an animal to reach the platform (latency) was measured. The daily improvement (in seconds to reach the hidden platform) for each animal (in comparison to the starting day) was evaluated.

### Elevated Plus-Maze (EPM)

The elevated plus maze (EPM) trial is used for testing anxiety, based on the assumption that animals suffer from fear of open spaces. The maze consists of two open arms and two closed arms (50 cm × 10 cm × 40 cm each). The arms of each type are opposite to each other. The maze is elevated to 50 cm height from the floor. Mice were placed onto the center of the maze, facing an open arm, and left free to explore it for 5 min. The time spent in the open and closed arms was recorded and compared. The data were analyzed using the following formula: D2 = (b − a)/(b + a), in which “a” designated the time spent in the open arms, and “b” designated the time spent in the closed arms (Alcalay et al., 2004). The longer stay in the closed arms reflects increased anxiety-like behavior (Pellow et al., 1985; Treit et al., 1993).

### Open Field

The open field apparatus is a 50 × 50 cm square arena, with 30 cm high walls (white/black colored). Mice were individually placed in the open field and left to explore it freely for 15 min. The distance moved and time spent in the entire open field, as well as in its inner defined quadrants (center, border) were measured.

### *In silico* Analysis

EB1 and EB3 homodimers (Honnappa et al., 2009; Bjelić et al., 2012) were used in order to predict the SKIP and D-SKIP conformations. Flexible docking was performed using Rosetta FlexPepDock (Raveh et al., 2010).

### Statistical Analysis

Results are presented as means ± standard error of the mean (SEM). For two different categorical independent variables, two-way analysis of variance (ANOVA; for the elevated plus maze and open field tests) or two-way repeated-measures ANOVA (for the MWM test), followed by Tukey *post hoc* test were performed. Exact *p*-values for main effects are stated throughout the manuscript, whereas exact *post hoc* *p*-values are stated in the legends, with values smaller than 0.05 considered significant. Non-significant *P*-values for main effects are stated in the figure legends. For all *in vivo* procedures, all data were taken into consideration for the statistical analyses, conducted using either SigmaPlot software version 11 Inc. for Windows (Chicago, IL, USA), or GraphPad Prism versions 6 and 8 Inc. for Windows (La Jolla, CA, USA).

### Study Approval

All procedures involving animals were conducted under the supervision and approval of the Animal Care and Ethics Committee of Tel Aviv University and the Israel Ministry of Health (M-15-059).

## Results

### *Adnp*^+/–^ Mice Display Spatial Learning Deficiencies in the MWM, With SKIP Providing Improvement, but Not D-SKIP

The MWM paradigm included two daily trials, aimed at assessing the impact of the *Adnp* genotype on spatial learning and memory abilities, as well as the effect of SKIP and D-SKIP. Latencies to find the hidden platform was measured daily, for 5 days, with the first daily trial measuring reference memory (trial 1), and the second daily trial evaluating short-term memory (trial 2; Gordon et al., 1995; Gozes et al., 2000a). Learning was defined as the latency to find the hidden platform on a given experimental day, compared with the latency to find the platform on the first day.

In daily trial 1 (reference memory, Figure 1A), main effects for group (*F*_(5,208)_ = 4.485, *p* = 0.002) and day (*F*_(4,208)_ = 9.124, *p* < 0.001) were found. Specifically, vehicle-treated *Adnp*^+/+^ mice learned the task on day 5 of the MWM, contrasting *Adnp*^+/–^ mice. SKIP-treated *Adnp*^+/–^ mice showed an unstable improvement on day 2, which was not observed on day 3, but significantly stabilized on days 4 and 5. D-SKIP did not show an effect on *Adnp*^+/–^ mice. In *Adnp*^+/+^ mice, while SKIP had no effect, D-SKIP-treatment showed a sporadic improvement on days 3–4, followed by an exacerbation on day 5.

**Figure 1:** Reference and short-term memory in the morris water maze (MWM): *Adnp*^+/+^ mice learn the task, whereas *Adnp*^+/–^ mice are impaired, with SKIP and D-SKIP displaying different behavioral outcomes. First and second daily water maze trials measuring reference and short-term memory are presented. To measure performance throughout the experimental days of the MWM, a two-way repeated-measures analysis of variance (ANOVA) with Tukey *post hoc* test was performed (*Adnp*^+/+^ *N* = 13; *Adnp*^+/+^ SKIP *N* = 7; *Adnp*^+/+^ D-SKIP *N* = 8; *Adnp*^+/–^ *N* = 12; *Adnp*^+/–^ SKIP *N* = 7; *Adnp*^+/–^ D-SKIP *N* = 11). The trials were implemented over five consecutive days. Latency measured in seconds to reach the hidden platform in its new daily location is depicted. **(A)** For Trial 1 [a non-significant value was observed for main interaction effect (*F*_(20,208)_ = 1.0301, *p* = 0.427)], Tukey *post hoc* tests showed that *Adnp*^+/+^ male mice learned the task on day 5 (*p = 0.034), compared with the impaired *Adnp*^+/–^ mice. D-SKIP treatment led to some improved performance on days 3–4 (*p = 0.040, **p = 0.008, respectively), which was then exacerbated on day 5. SKIP-treated *Adnp*^+/–^ mice learned the task on days 2, 4–5 (**p = 0.003, **p = 0.009, *p = 0.034, respectively). **(B)** For Trial 2 [a non-significant value was observed for main interaction effect (*F*_(20,208)_ = 1.119, *p* = 0.332)], Tukey *post hoc* effects showed that vehicle-treated *Adnp*^+/+^ male mice learned the task on days 4–5 (**p = 0.003, ***p < 0.001, respectively), compared with the impaired *Adnp*^+/–^ mice. SKIP-treated *Adnp*^+/+^ mice learned the task on days 4–5 (**p = 0.004, **p = 0.008, respectively). On day 5, a significant difference was found between SKIP- and D-SKIP treated *Adnp*^+/–^ mice (^##^*p* = 0.006).

In daily trial 2 (short-term memory, Figure 1B), main effects for group (*F*_(5,208)_ = 4.303, *p* = 0.002) and day (*F*_(4,208)_ = 10.453, *p* < 0.001) were found. Vehicle- and SKIP-treated *Adnp*^+/+^ mice learned the task on days 4–5 of the MWM task, as opposed to *Adnp*^+/–^ mice. Also, on day 5, a significant difference was found between SKIP- and D-SKIP treated *Adnp*^+/–^ mice, with D-SKIP mice taking about 3-fold more time to find the hidden platform compared to SKIP-treated mice.

### SKIP and D-SKIP Lead to Distinctive Anxiety-Related Behavioral Outcomes in the EPM and Open Field Tests

To evaluate anxiety-related behavior, the EPM and the open field behavioral tests were implemented. In the EPM test (Figure 2A), main effects for genotype (*F*_(1,90)_ = 6.242, *p* = 0.014) and treatment (*F*_(2,90)_ = 21.109, *p* < 0.001) were found. Specifically, SKIP-treated *Adnp*^+/+^ mice spent significantly more time in the closed arms, compared with the vehicle- and D-SKIP-treated groups. In *Adnp*^+/–^ mice, SKIP-treated animals spent significantly more time in the closed arms, compared with the D-SKIP-treated group only. In contrast, D-SKIP-treated *Adnp*^+/+^ and *Adnp*^+/–^ mice spent more time in the open arms, compared with vehicle-treated control groups, thus indicating a possible altered anxiety-related/increased risky behavior.

**Figure 2:** SKIP treatment ameliorates the behavior of *Adnp*^+/–^ male mice in the elevated plus-maze and open field, whereas D-SKIP aggravates. Two-way ANOVA with Tukey *post hoc* test was performed (*Adnp*^+/+^ *N* = 16–22; *Adnp*^+/+^ SKIP *N* = 10–17; *Adnp*^+/+^ D-SKIP *N* = 8; *Adnp*^+/–^ *N* = 13–20; *Adnp*^+/–^ SKIP *N* = 9–16; *Adnp*^+/–^ D-SKIP *N* = 12–13). **(A)** Elevated plus maze [EPM; A non-significant value was observed for main interaction effect (*F*_(2,90)_ = 0.953, *p* = 0.389)]: In *Adnp*^+/+^ mice, SKIP-treated animals spent more time in the closed arms, compared with their D-SKIP- and vehicle-treated counterparts. In *Adnp*^+/–^ mice, D-SKIP-treated animals spent more time in the open arms, compared with SKIP- and vehicle-treated mice. In *Adnp*^+/+^ mice, significant Tukey *post hoc* differences were observed between SKIP- and both vehicle- and D-SKIP-treated mice (**p = 0.002, ***p < 0.001, respectively). In *Adnp*^+/–^ mice, significant differences were observed between SKIP- and D-SKIP-treated mice (***p < 0.001), as well as between D-SKIP- and vehicle-treated mice (*p = 0.028). **(B)** Open field—Total Distance Traveled [non-significant values for main effects included genotype (*F*_(1,63)_ = 0.467, *p* = 0.497) and interaction (*F*_(2,63)_ = 0.845, *p* = 0.434) effects]: SKIP-treated *Adnp*^+/+^ mice traveled a decreased distance, compared with their D-SKIP- and vehicle-treated counterparts. In addition, D-SKIP-treated *Adnp*^+/–^ mice displayed an increased distance, compared with SKIP- and vehicle-treated mice. In *Adnp*^+/+^ mice, significant Tukey *post hoc* differences were observed between SKIP- and both vehicle- and D-SKIP-treated mice (**p = 0.008, ***p < 0.001, respectively). In *Adnp*^+/–^ mice, significant differences were observed between SKIP- and D-SKIP-treated mice (**p = 0.002), as well as D-SKIP- vs. vehicle-treated mice (*p = 0.033). **(C)** Open field—Duration in Center Zone [non-significant values for main effects included genotype (*F*_(1,62)_ = 2.458, *p* = 0.122), treatment (*F*_(2,62)_ = 0.0601, *p* = 0.942) and interaction effects (*F*_(2,62)_ = 0.408, *p* = 0.667)]: no significant *post hoc* differences were observed between the experimental groups.

In the open field test (Figure 2B), the total distance traveled/locomotor activity was measured in all experimental groups, with a main treatment effect found (*F*_(2,63)_ = 17.889, *p* < 0.001). This parameter has been previously linked with positive symptoms of schizophrenia, and general psychotic behavior (van den Buuse et al., 2005; Merenlender-Wagner et al., 2010, 2014; van den Buuse, 2010). While no genotype-related phenotype was shown, SKIP-treated mice of both genotypes traveled a significantly decreased distance, compared with vehicle- and D-SKIP-treated groups, as in the case of *Adnp*^+/+^ mice, or D-SKIP-treated group only, as in the case of *Adnp*^+/–^ mice. Furthermore, D-SKIP-treated *Adnp*^+/+^ and *Adnp*^+/–^ mice traveled a longer distance, compared with the vehicle-treated control groups. When looking at the time spent in the center zone of the open field arena (Figure 2C), no significant differences were observed between the experimental groups.

### SKIP and D-SKIP Interact With EB1 and EB3 Proteins in Distinctive Conformations

*In silico* analysis showed that the four-amino-acid peptides SKIP and D-SKIP bind EB1 and EB3 proteins using different residues, thus resulting in distinctive binding conformations. Specifically, in EB1, SKIP binds Tyrosine 217 (Y217), whereas D-SKIP binds Arginine 222 (R222; Figure 3A). Furthermore, in EB3, SKIP binds Glutamate 225 (E225), but D-SKIP does not (Figure 3B).

**Figure 3:** SKIP and D-SKIP bind in silico EB1 and EB3 in distinct conformations. Three-dimensional (3D) structures of EB1 and EB3 homodimers (green and cyan) are shown as ribbons. SKIP (yellow) and D-SKIP (purple) peptides are shown as sticks. **(A)** In EB1, SKIP binds Tyrosine 217 (Y217), whereas D-SKIP binds Arginine 222 (R222). **(B)** In EB3, SKIP binds Glutamate 225 (E225), but D-SKIP does not. The figures were generated using Pymol. The best scoring conformations are shown.

## Discussion

The current study has examined *in vivo* cognitive and anxiety-related behavioral aspects in the unique *Adnp*-haploinsufficient mouse model, when treated with either SKIP or D-SKIP peptides, both derived from the ADNP-snippet, NAP. The results indicated that *Adnp* deficiency impairs the cognitive state of the animals, and that this condition may be ameliorated by SKIP treatment, but not by D-SKIP. It should be noted that the study was performed on relatively aged animals, with treatment beginning at the age of 6 months, and behavioral tests performed at the age of 7–9 months. In this respect, the *Adnp*-deficient phenotype was previously shown to present increased age-dependent neurodegeneration and tauopathy (Vulih-Shultzman et al., 2007; Hacohen-Kleiman et al., 2018). This phenotype can also be explained by the highly important role of ADNP as vital for mammalian brain formation and function (Pinhasov et al., 2003; Vulih-Shultzman et al., 2007), and as a master-gene regulating hundreds of key genes (Vulih-Shultzman et al., 2007; Amram et al., 2016). Interestingly, with PACAP, known to regulate ADNP (Zusev and Gozes, 2004), various similarities were observed between the *Adnp*-haploinsufficient mouse model and PACAP-deficient mice. These included slower weight gain during the first weeks of life, coupled with delayed neurobehavioral development (Farkas et al., 2017; Hacohen-Kleiman et al., 2018). Furthermore, dentition in old and young mice was associated with PACAP (Sandor et al., 2014, 2016), while tooth eruption in mice and children was associated with ADNP (Gozes et al., 2017b).

In terms of cognition, the evaluation of the *Adnp*-haploinsufficient mouse model by the MWM paradigm corroborated previous findings in male *Adnp*^+/–^ mice, exhibiting spatial learning deficiencies (Vulih-Shultzman et al., 2007). The current results with SKIP in the MWM are supported by previous social behavioral tests, coupled with the social/olfactory abilities improved by SKIP, but not D-SKIP (Amram et al., 2016). The results are also supported by past findings with the parent peptide NAP, showing significant improvement in learning the MWM task (Vulih-Shultzman et al., 2007). Altogether, these findings provide evidence for the neuroprotective nature of SKIP, but not D-SKIP. Importantly, while the MWM test may partially rely on visual cues, mice are not considered “visual animals,” but rather nocturnal, relying primarily on olfactory and auditory cues as well as touch/balance senses (use of whiskers for sensing the environment; Pinto and Enroth-Cugell, 2000). Specifically, the ICR background strain of the *Adnp*-deficient mouse model used here, as well as white mice, in general, may suffer retinal abnormalities, causing reduced visual abilities (Keeler, 1924). However, the degree of visual impairment is not the same within all albino mice (Wong and Brown, 2006). It should also be noted that for the MWM task, ICR mice were utilized before in multiple independent studies (Ge et al., 2013; Wang et al., 2014; Kim et al., 2015; Kitanaka et al., 2015).

An additional aspect examined was anxiety-related behavior, by implementing the EPM and open field behavioral tests. In the EPM, D-SKIP opposed the effects of SKIP, thus leading to a reduced anxiety-like phenotype and an increased altered/risky behavior. A similar finding was previously found in PACAP- and PAC1 receptor-null mice, thereby implying that the ADNP-regulating PACAP, plays a role in stress mechanisms (Hammack et al., 2009; Vaudry et al., 2009). In the open field test, SKIP led to a hypo-locomotive behavior, suggesting an increased anxiety-like state (Coelho et al., 2014; Park et al., 2018). This correlates the finding observed in SKIP-treated mice in the EPM (increased D2 score indicating an increased anxiety level), preserving a normal mouse phenotype. However, the effect of D-SKIP treatment contrasted SKIP, with a significantly increased total distance traveled (hyper-locomotion), previously linked with psychotic behavior (van den Buuse et al., 2005; Merenlender-Wagner et al., 2010, 2014; van den Buuse, 2010), compared with vehicle- and SKIP-treated mice. This finding of D-SKIP-treated mice being hyperactive in the open field could also offer a possible explanation to the reference memory result in the MWM, where it may seem that D-SKIP first improved and finally worsened reference memory in *Adnp*^+/+^ mice. Importantly, there may be additional factors affecting open-field behavior (e.g., locomotor activity) including sex, strain and stress (Sestakova et al., 2013). In this respect, we have previously shown an increased locomotor activity in *Adnp*^+/–^ female mice. This behavior was exacerbated by stress-challenge, with a further significant increase in locomotion, partially ameliorated by PACAP (Sragovich et al., 2019b). To summarize our mouse behavioral findings, it should be noted that there may be some data variability in this type of experiment, thus posing a certain limitation. Nevertheless, all the *in vivo* experiments implemented in the current study, have shown that the most highly repeated significant findings were the opposite phenotypic outcomes observed in SKIP- and D-SKIP-treated mice. Combined with rigorous statistical analyses, the validity of these experimental findings was confirmed.

Complementing the above *in vivo* behavioral results, a bioinformatics *in silico* analysis has suggested that SKIP and D-SKIP, both containing the SIP motif, which serves as the NAP EB binding site (Oz et al., 2014; Amram et al., 2016), interact with the tubulin/microtubule EB1 and EB3 proteins in distinctive conformations. The different *in silico* binding patterns observed between SKIP and D-SKIP to EB1/EB3 conform to the different interaction patterns previously found between these two peptides and NAP in NMR analysis, with SKIP, but not D-SKIP, interacting with NAP (Amram et al., 2016). Interestingly, a follow-up NMR analysis displayed an interaction between NAP and the neuroprotective peptide D-SAL (Gozes et al., 2016). This finding suggested a possible potential direct interaction of D-SAL with the endogenous ADNP, to provide microtubule fortification and neuroprotection, as was also previously shown *in vivo* (Shiryaev et al., 2011). Importantly, the protection by SKIP was thoroughly described from the *in vitro* level, in a cell culture model of zinc intoxication, to the *in vivo* social behavior and histological levels (Amram et al., 2016). This has proven that it is based on the NAP core sequence, and despite being shortened by half, the 4-amino-acid SKIP did not result in a loss of function (Amram et al., 2016). Furthermore, *in vitro* binding experiments performed for the neuroprotective parent peptides NAP (NAPVSIPQ) and NAPVSKIPQ, have shown an interaction with EB1/EB3, thus enhancing synaptic plasticity (Oz et al., 2014). When using affinity chromatography, SKIP was shown to enhance the interaction of the NAPVSIPQ motif of Adnp with EB3, suggesting augmentation of Adnp MT fortification under compromised situations, such as *Adnp* haploinsufficiency (Amram et al., 2016). NAP and SKIP were also shown to increase microtubule dynamics, through a mechanism of EB1/EB3 and Tau recruitment to microtubules, thereby providing neuroprotection (Ivashko-Pachima et al., 2017; Ivashko-Pachima and Gozes, 2019). Therefore, our findings may partially explain the distinctive natures of SKIP and D-SKIP, possibly underlying the *in vivo* behavioral outcomes presented in the current study. Importantly, it should be kept in mind that despite the increased accessibility of *in silico* technologies to scientists, allowing the enhancement of drug development processes, these are essentially predictive methods, the results of which should be interpreted cautiously (Valerio, 2009).

To conclude, as was previously shown (Amram et al., 2016), and here as well, binding inhibition may be caused in the case of SKIP, when replacing the L-amino-acids with D-amino-acids. Furthermore, it is possible that SKIP and D-SKIP mediate distinct actions in the brain. In this respect, we have previously shown in the hippocampus that the SKIP normalized the expression of the ASD-linked gene *Slc6a4*, encoding a serotonin transporter, whereas D-SKIP did not, thus providing a partial explanation to the distinctive *in vivo* behavior (Amram et al., 2016). Since the NAP-derived SKIP was previously presented as a novel future therapeutic option for potential ASD drug development (Amram et al., 2016), the current findings are of great importance. This is also in light of our recent results, showing that the *Adnp*^+/–^ mouse mimics the human autism-like *ADNP* syndrome patient, and suggesting NAP as a drug candidate for treating this pathology (Hacohen-Kleiman et al., 2018). Therefore, the present study has practical pharmacological significance, as it is important to distinguish between agonists and antagonists, thus assisting at making crucial therapeutic decisions at an early stage of the drug development process.

## Data Availability Statement

The datasets generated for this study are available on request to the corresponding author.

## Ethics Statement

The animal study was reviewed and approved by the Animal Care and Ethics Committee of Tel Aviv University and the Israel Ministry of Health (M-15-059).

## Author Contributions

SS provided input to project design, performed experiments, analyzed data, and wrote the article. NA performed experiments and analyzed data. AY performed the bioinformatics *in silico* analysis. Prof. IG led the entire project, provided funding, designed experiments, analyzed data, and wrote the article.

## Conflict of Interest

IG is the Chief Scientific Officer of Coronis Neurosciences. NAP (CP201) use is under patent protection (US patent nos. US7960334, US8618043, and USWO2017130190A1). The remaining authors declare that the research was conducted in the absence of any commercial or financial relationships that could be construed as a potential conflict of interest.
